RETRACTED

# Prediction and optimization of employee turnover intentions in enterprises based on unbalanced data

**DOI:** 10.1371/journal.pone.0290086

**Published:** 2023-08-17

**Authors:** Zhaotian Li, Edward Fox

**Affiliations:** 1 Metropolitan College, Boston University, Boston, Massachusetts, United States of America; 2 Department of Computer Science, Virginia Tech, Arlington, Virginia, United States of America; St Xavier’s Catholic College of Engineering, INDIA

## Abstract

The sudden resignation of core employees often brings losses to companies in various aspects. Traditional employee turnover theory cannot analyze the unbalanced data of employees comprehensively, which leads the company to make wrong decisions. In the face the classification of unbalanced data, the traditional Support Vector Machine (SVM) suffers from insufficient decision plane offset and unbalanced support vector distribution, for which the Synthetic Minority Oversampling Technique (SMOTE) is introduced to improve the balance of generated data. Further, the Fuzzy C-mean (FCM) clustering is improved and combined with the SMOTE (IFCM-SMOTE-SVM) to new synthesized samples with higher accuracy, solving the drawback that the separation data synthesized by SMOTE is too random and easy to generate noisy data. The kernel function is combined with IFCM-SMOTE-SVM and transformed to a high-dimensional space for clustering sampling and classification, and the kernel space-based classification algorithm (KS-IFCM-SMOTE-SVM) is proposed, which improves the effectiveness of the generated data on SVM classification results. Finally, the generalization ability of KS-IFCM-SMOTE-SVM for different types of enterprise data is experimentally demonstrated, and it is verified that the proposed algorithm has stable and accurate performance. This study introduces the SMOTE and FCM clustering, and improves the SVM by combining the data transformation in the kernel space to achieve accurate classification of unbalanced data of employees, which helps enterprises to predict whether employees have the tendency to leave in advance.

## Introduction

With the economic development and the industry transformation, how to attract and retain talents is crucial to the development of enterprises [1]. The departure of employees, especially the core employees, often brings losses to the company in various aspects. Employee departures can cause costly damage to the company, as well as negative emotional impact on other employees [2, 3]. The departure of core employees can cause the enterprise to lose its core technology or important customers, which is irretrievable for the enterprises [4]. At present, many companies have established datasets that can be used to predict the tendency of employees turnover through statistics, surveys and questionnaires for HR and other departments to analyze and introduce relevant policies to to retain employees, such as salary, culture, emotion, etc [5].

RETRACTED

Traditional employee turnover theories tend to analyze and compare only a small portion of employee data, and cannot fully analyze the collected employee information data comprehensively, which may lead to inaccurate results and cause companies to make wrong decisions in the end [6, 7]. At the same time, there is a large amount of unbalanced data with widely varying sample sizes in real life, such as medical pathology diagnosis, credit card fraud, network intrusion information, business operations and employee turnover data [8, 9]. The traditional Support Vector Machine (SVM) can lead to the resulting hyperplane being more biased toward minority class, making them misclassified as majority class. Therefore, how to improve the recognition rate and overall performance of minority class in unbalanced data is the important research topic in the field of machine learning [10–12].

Developed countries in the West have long been analyzing and studying the relationship between enterprises and employees, including employee performance and employee turnover [13]. Employee turnover, as one of the core of enterprise research, has been the subject of research in resource management, social behavior, and employee mobility theories [14]. At present, many scholars have proposed a series of theoretical models of employee turnover by collecting data on employees’ work situation and satisfaction. These data are usually simplified into work reward, work environment, corporate culture and work group [15]. These four dimensions are used to model the relationship between employee turnover and corporate strategies to help companies improve employee satisfaction and reduce turnover. Marquardt D J [16] suggested that the relationship between leaders and employees has a strong relationship on whether employees want to stay in the company for a long time. The harmonious relationship will lead to more tacit understanding among the company’s employees at work. Leaders can motivate their employees to work in a motivating way to improve their work efficiency. Berber N [17] proposed a model of employee satisfaction based on career values, analyzing employees’ satisfaction with the company and career value. Khairunisa N A [6] accurately measured the relationship between the probability of employees leaving their jobs, the amount of effort they put into their jobs, and the level of support from the company. Kasdorf R L [18] used structural equation modeling to analyze the relationship between company fairness and employee turnover, and proposed the mechanism to influence company fairness and employee turnover.

RETRACTED

Nowadays, most companies pay more attention to questionnaire research and information collection for employees. Therefore, analyzing employee data through SVM algorithm and building employee turnover model with existing samples can more effectively enable companies to detect employee turnover earlier [7, 10]. There are many mature SVM algorithms that have very good classification results when facing balanced samples. However, in datasets with unbalanced samples, SVM algorithms often misclassify the minority class into the majority, constituting the sample defect in unbalanced datasets, which leads to encountering problems such as sample scarcity [19], boundary ambiguity [20], and noise pollution [21].

Traditional data sampling methods can lead to overfitting of the datasets and loss of important feature information in the classification model. Therefore, Pei W [22] proposed the Synthetic Minority Oversampling Technique (SMOTE) based on the analysis of the proximity between sample points to synthesize the minority class; then, they [23] proposed the feature selection method to solve the problem of high-dimensional unbalanced datasets. By analyzing the intrinsic relationships existing between samples through non-random sampling, the original feature information is maintained in the sampling process, making the classification model less prone to overfitting and misclassification during the training process [24, 25]. Cost-sensitive learning reduces the error of SVM in classifying minority classes by reducing the overall cost of misclassification and improves the classification of unbalanced data [26]. Vanderschueren T [27] improved the general learning model into the cost-sensitive learning model by calculating the ideal cost for each sample and modifying the original sample class to obtain the new sample set. Ren Z [28] used fuzzy learning to reduce the effect of noise in samples on classification and combined the cost-sensitive mechanism to reduce the sensitivity of unbalance distribution. Li J [29] combined AdaBoost and sample generation techniques to regenerate new majority and minority class samples. Zhou B [30] improved the weight update rule of the Boosting algorithm and introduced a misclassification cost mechanism to improve the accuracy. Liu J [31] proposed the random forest algorithm with weights, introduced weighting techniques in the construction of decision trees, and used voting with weights in the decision process to improve the prediction ability. The feature selection method represents the objects in the original dataset with a subset of features and removes redundant feature information [32]. Parlak B [33] extracted more representative and discriminative features, which effectively improved the classification accuracy. Nurhasanah R [34] proposed Feature Assessment by Sliding Thresholds (FAST) to evaluate feature subsets and feature classifiers based on ROC curve area.

RETRACTED

The SMOTE is introduced to improve the shortcoming of SVM (SMOTE-SVM) for newly generated samples without misclassification cost in the classification process. The improved FCM clustering is proposed to generate new samples in combination with the SMOTE (IFCM-SMOTE-SVM), which greatly reduces the chances of noisy data generation. Using the kernel function of SVM to transform the data into a high-dimensional feature space before clustering and sampling, a kernel space-based classification algorithm (KS-IFCM-SMOTE-SVM) is obtained, and the method is experimentally demonstrated to have a great improvement on the SVM classification. The researches of the paper have a good practical value and application prospect in turnover prediction and employee management.

### Classification of unbalanced data based on SMOTE-SVM

#### Prediction principle of employee turnover based on SVM

Assuming that the sample set of employee information is $\{\left(x_{1},y_{1}),\ldots ,(x_{i},y_{i}),\ldots ,(x_{n},y_{n}\right)\},i=1,\ldots ,n$, where *n* represents the number of employees in the enterprise, *x*_*i*_∈*R*^*m*^, and *m* represents the information dimension; the classification label is *y*_*i*_ = {−1,+1}, where -1 represents the resigned employees and +1 represents the active employees. On the *R*^*n*^ space, a real number function *g*(*x*) = (*W*^*T*^*x*+*b*) that minimizes the classification boundary $\frac{1}{2}\|w{\|}^{2}$ is found so as to determine the classification decision plane of whether an employee leaves or not, and finally the decision function *f*(*x*) = sgn(*g*(*x*)) is used to predict the category of whether a new employee leaves or not.

For the simple low-dimensional employee dataset, SVM can obtain the maximum interval plane by solving the following problem:

$$\begin{array}{c} \min\frac{1}{2}\|w{\|}^{2}\\ s.t.\;y_{i}(W^{T}x_{i}+b)\geq +1\\ i=1,\ldots ,n \end{array}$$ (1)

To transform the solution problem by Lagrange pairwise method:

$$L(\alpha ,w,b)=\frac{1}{2}\|w{\|}^{2}-\sum_{i=1}^{n}\alpha_{i}[y_{i}(W^{T}x_{i}+b)-1]$$ (2)

Where *α*_*i*_ ≥ 0 is the Lagrange multiplier. Eq (2) can be transformed into pairwise problem:

$$\begin{array}{c} \max_{\alpha }L(\alpha )=\sum_{i=1}^{n}\alpha_{i}-\frac{1}{2}\sum_{i=1}^{n}\sum_{j=1}^{n}\alpha_{i}\alpha_{j}y_{i}y_{j}x_{i}x_{j}\\ s.t.\sum_{i=1}^{n}y_{i}\alpha_{i}=0,\alpha_{i}\geq 0 \end{array}$$ (3)

The hyperplane function of the classification decision can be obtained after solving:

$$f(x)=w^{T}x+b=\sum_{i=1}^{n}\alpha_{i}y_{i}x_{i}^{T}x+b$$ (4)

Since the samples are disturbed by noise, the data are not linearly differentiable, which has a great impact on the training results of the SVM. The relaxation variable *ξ*_*i*_ (*ξ*_*i*_ > 0), an allowable deviation function interval, is introduced, and the corresponding optimization objective becomes:

$$\begin{array}{c} \min\frac{1}{2}\|w{\|}^{2}+C\sum_{i=1}^{n}\xi_{i}\\ s.t.y_{i}(w^{T}x_{i}+b)\geq 1-\xi_{i}\\ \xi_{i}>0,i=1,\ldots ,n \end{array}$$ (5)

Where *C* is the penalty factor, *α*_*i*_ < *C*.

RETRACTED

For the higher dimensional, linearly indistinguishable employee information, the above approach cannot be used to find the optimal classification plane. Therefore, SVM projects the original nonlinear employee mapping function *φ* into the high-dimensional space. In the high-dimensional feature space, the employee datasets will become linearly separable and can be solved linearly. With the introduction of the mapping function, the form of the solution function becomes:

$$\begin{array}{c} \min\frac{1}{2}\|w{\|}^{2}+C\sum_{i=1}^{n}\xi_{i}\\ s.t.y_{i}(w\cdot \varphi (x_{i})+b)\geq 1-\xi_{i}\\ \xi_{i}>0,i=1,\ldots ,n \end{array}$$ (6)

As in the linear solution approach, the solution of the original equation needs to be obtained by solving the pairwise problem:

$$\begin{array}{c} \min\frac{1}{2}\sum_{i=1}^{n}\sum_{j=1}^{n}y_{i}y_{j}\alpha_{i}\alpha_{j}k(x_{i}\cdot x_{j})-\sum_{j=1}^{n}\alpha_{j}n\\ s.t.\sum_{i=1}^{n}y_{i}\alpha_{j}=0,0\leq \alpha_{i}\leq C \end{array}$$ (7)

Where *α*_*i*_ is the Lagrange multiplier; *k*(*x*_*i*_⋅*x*_*j*_) is the kernel function, and $k(x_{i}\cdot x_{j})=\varphi (x_{i})\cdot \varphi (x_{j})$. The special solution α* of the Lagrange multiplier is obtained by solving, and the weight vector is calculated, i.e:

$$w^{*}=\sum_{i=1}^{n}\alpha^{*}y_{i}\varphi (x_{i})$$ (8)

Then the threshold b* is calculated in two cases:

(1) If 0 < *α*_j_* < *C* exists, a positive component *α*_j_* of α* is chosen and calculated:

$$b^{*}=y_{j}-\sum_{i=1}^{n}\alpha^{*}y_{i}k(x_{i}\cdot x_{j})$$ (9)

(2) If 0 < *α*_j_* < *C* does not exist, i.e., the component of α* is 0 or *C*, then the range of b* is [*b*_min_+*b*_max_]. In the actual calculation, generally *b* takes the middle value, i.e:

$$b^{*}=\frac{b_{\min}+b_{\max}}{2}$$ (10)

The final constructed decision function is:

$$f(x)=\mathrm{sgn}(\sum_{i=1}^{n}\alpha^{*}y_{i}k(x_{i}\cdot x_{j})+b^{*})$$ (11)

#### Cost-sensitive weighting-based classification of unbalanced data

From the above, the traditional SVM has better performance when the number of two class samples are approximately the same. However, when the datasets are unbalanced, the classification performance of SVM is greatly reduced. In the problem of classifying the turnover intention of employees, especially in larger companies, the number of employee turnover is generally a small percentage of employees. The prediction result of SVM often incorrectly classifies employees with turnover intention into active employees, which leads to inaccurate judgment of turnover intention. This paper firstly introduces the SMOTE algorithm, which randomly selects the neighboring data of the original data and manually synthesizes the new samples between the original and neighboring data, so that the data of resigned employees and active employees can reach the balance.

RETRACTED

The sample *x*_*i*_ is randomly selected in the sample set of resigned employees, and then a sample *x*_*j*_ of resigned employees is randomly selected from the neighborhood data, and finally the new sample is synthesized by the following equation:

$$x_{new}=x_{i}+rand(0,1)\times (x_{i}-x_{j})$$ (12)

The SMOTE does not consider the effect of noise when synthesizing data, which can lead to the synthesized data increasing the noise rate of the original samples and affecting the accuracy of the SVM. Therefore, this paper proposes the SMOTE-SVM based on the cost-sensitive weighting for minority classes, majority classes, and synthetic instances with different weighting [35]. The original optimization function is as follows:

$$\begin{array}{c} \min_{w,b,\xi }\frac{1}{2}w^{T}w+C\times k^{maj}\sum_{i=1}^{\left|s^{majj}\right|}\xi_{i}^{maj}+C\times k^{\min}\sum_{i=1}^{\left|s^{\min}\right|}\xi_{i}^{\min}+C\times k^{syn}\sum_{i=1}^{\left|s^{syn}\right|}\xi_{i}^{syn}\\ s.t.w^{T}\varphi (x_{i})+b\leq 1-\xi_{i}^{maj}\;\forall x_{i}\in S^{maj}\\ w^{T}\varphi (x_{i})+b\leq 1-\xi_{i}^{\min}\;\forall x_{i}\in S^{\min}\\ w^{T}\varphi (x_{i})+b\leq 1-\xi_{i}^{syn}\;\forall x_{i}\in S^{syn}\\ \xi_{i}^{maj},\xi_{i}^{\min},\xi_{i}^{syn}\geq 0 \end{array}$$ (13)

Where the weight factors *c*^*maj*^, *c*^*min*^, and *c*^*syn*^ control the misclassification cost of the majority class, minority class, and synthetic instances, respectively. The method allows the SVM to control the separation hyperplane more finely by weighting the instances differently [36]. The obtained α* is used to determine the class *y* of the new instance *α*_*new*_:

$$y=sign\{\sum_{i=1}^{\left|S\right|}a_{i}^{*}y_{i}K(x,x_{i})+\sum_{i=1}^{\left|S^{syn}\right|}a_{i}^{*}K(x,x_{i}^{pq})+b$$ (14)

The experimental comparison of multiple sets of unbalanced data reveals that the cost-sensitive weighted SMOTE-SVM has some improvement in classification accuracy and also reduces the risk of overfitting compared to SVM for unbalanced data.

RETRACTED

### Sampling of unbalanced data based on fuzzy C-mean clustering

#### Clustering of resigned employees based on fuzzy C-mean (FCM)

The FCM first fuzzes the datasets of departing employees, and then divides the datasets. To determine the degree of affiliation of each data point, the affiliation value in the range [0,1] is used to assign the value to the data points. Constraints within this affiliation range are also needed to normalize the affiliation matrix such that the affiliation of the data points to each category sums to 1:

$$\sum_{i=1}^{c}u_{ij}=1,\;\forall j=1,\cdots ,n$$ (15)

The general equation of the objective function of FCM is:

$$J_{m}(U,P)=\sum_{i=1}^{c}\sum_{j=1}^{n}u_{ij}^{m}d_{ij}^{2}$$ (16)

Where the value of *u*_*ij*_ is the real number between 0, 1; *m* is a weighted index greater than 1, which is the fuzzy indicator [37]. The new objective function is constructed using the Lagrange multiplier and Eqs (15) and (16) as follows:

$$\begin{array}{l} J(U,P,\lambda_{1},\cdots ,\lambda_{n})=J(U,P)+\sum_{j=1}^{n}\lambda_{j}\left(\sum_{i=1}^{c}u_{ij}-1\right)\\ \;=\sum_{i=1}^{c}\sum_{j=1}^{n}u_{ij}^{m}d_{ij}^{2}+\sum_{j=1}^{n}\lambda_{j}\left(\sum_{i=1}^{c}u_{ij}-1\right) \end{array}$$ (17)

Where *λ*_*j*_, *j* = 1,⋯,*n* is the Lagrange multiplier of the *n* constraint of Eq (15), so the solutions of Eqs (15), (16) and (17) are equivalent [37]. By taking partial derivatives of all parameters so that the result is zero, the condition is obtained as:

$$c_{i}=\frac{{\sum_{j=1}^{n}u_{ij}}^{m}x_{j}}{{\sum_{j=1}^{n}u_{ij}}^{m}}\;and\;u_{ij}=\frac{1}{\sum_{k=1}^{c}{\left(\frac{d_{ij}}{d_{kj}}\right)}^{2/(m-1)}}$$ (18)

Where *c*_*i*_ is the clustering center matrix; *u*_*ij*_ is the fuzzy division matrix; *m* is a fuzzy indicator (*m* = 2), which is essentially a parameter that portrays the degree of fuzzification.

In order to obtain the clustering center of the resigned employees and the corresponding fuzzy affiliation value, so after determining the parameters of the FCM clustering by Eqs (17) and (18), the alternating iteration algorithm is then used to solve:

**Step 1**: Since the classes of resigned employees is greater than 2, it is assumed that the classes of resigned employees is *r* (2 ≤ *r* ≤ *n*), the number of resigned employees is *n*, the fuzzy index is *m* = 2, and the iteration threshold is *ε*, *ε* ∈ (0.001,0.01); the cluster center matrix of resigned employees is set as *P* ^(*t*)^, and *t* starts from 0.

RETRACTED

**Step 2**: The distance *d*_*ij*_^(*t*)^ from the sample of departing employees *x*_*j*_ to each sample center *c*_*i*_ is calculated [38]. The fuzzy division matrix is then updated after each calculation using Eq (18):

$$u_{ij}{}^{\left(t\right)}=\frac{1}{\sum_{k=1}^{c}{\left(\frac{d_{ij}{}^{\left(t\right)}}{d_{kj}{}^{\left(t\right)}}\right)}^{2/(m-1)}}$$ (19)

**Step 3**: The clustering center *P*^(*t+*1)^ is updated according to Eq (18), which then:

$$c_{i}=\frac{\sum_{j=1}^{n}{\left[u_{ij}{}^{\left(t\right)}\right]}^{m}x_{j}}{\sum_{j=1}^{n}{\left[u_{ij}^{\left(t\right)}\right]}^{m}}$$ (20)

**Step 4**: For a given threshold *m*, stop the iteration if $\|P^{\left(t+1\right)}-P^{\left(t\right)}\|\leq \varepsilon$, or if the iteration number exceeds the maximum number, otherwise let *t* = *t* + 1 and go to **Step 2**.

After the process is terminated, for each employee sample *x*_*j*_, the fuzzy clustering center and affiliation division matrix of the resigned employees are obtained. Eventually, the class to which the resigned employees can be determined:

$$k=\arg_{i=1,\cdots ,c}\max_{ij}$$ (21)

### Classification based on the improved FCM-SMOTE-SVM

Through the preliminary analysis of the data of the resigned employees, it is found that the data will be clustered near certain data. This is because the reasons for resigned employees tend to be related to each other. For example, employees who leave due to high work pressure have little time to travel to relax themselves, and also have aversion to work, etc. Therefore, this paper improves the FCM algorithm to first cluster the minority class of datasets, and then generate the new samples by SMOTE.

Assuming that the fuzzy classification matrix of the samples *X* = {*x*_1_,*x*_2_,⋯,*x*_*n*_} of resigned employees is *A* = [*u*_*ij*_]_*cxn*_, and the clustering center of resigned employees is *C* = [*c*_1_,*c*_2_,⋯,*c*_*n*_]^*T*^, as follows:

$$\{\begin{array}{c} \min\{J(A,c_{1},c_{2},\cdots ,c_{n})\}={\sum_{i=1}^{c}\sum_{j=1}^{n}a_{ij}}^{m}d_{ij}{}^{2}\}\\ s.t.\sum_{i=1}^{c}u_{ij}=1,\forall j=1,\cdots ,n \end{array}$$ (22)

Considering that the FCM clustering cannot accurately determine the classes of resigned employees and is more sensitive to the spatial distribution of clustered samples and noisy data. Therefore, we improved the FCM algorithm (IFCM) for clustering the samples [39]. The objective function of the IFCM algorithm is:

$$J_{IFCM}=\sum_{i=1}^{c}\sum_{j=1}^{n}{\left(u_{ij}\right)}^{m}\{1-\exp(-\beta {\left\|x_{j}-Z_{i}\right\|}^{2})\}$$ (23)

Where *u*_*ij*_ is the affiliation degree and *Z*_*i*_ is the new sample aggregation center:

$$u_{ij}=\frac{1/{\left[1-\exp(-\beta {\left\|x_{j}-z_{i}\right\|}^{2})\right]}^{1/(m-1)}}{\sum_{k=1}^{c}1/{\left[1-e(-\beta {\left\|x_{j}-z_{i}\right\|}^{2})\right]}^{1/(m-1)}}(i=1,2,\cdots ,n)$$ (24)

$$Z_{i}=\frac{\sum_{j=1}^{n}\left(u_{ij}\right)\exp(-\beta {\left\|x_{j}-z_{i}\right\|}^{2})x_{j}}{\sum_{j=1}^{n}{\left(u_{ij}\right)}^{m}\exp(-\beta {\left\|x_{j}-z_{i}\right\|}^{2})}\;(i=1,2,\cdots ,c)$$ (25)

The above method is combined with the SMTOE to pre-process the data of resigned employee to reduce the unbalanced samples, and also to improve the problem of excessive randomness that occurs in new samples synthesized randomly, as shown in Fig 1:

**Fig 1:** IFCM-SMOTE flow.

RETRACTED

The improved interpolation formula is:

$$X_{new}=Z_{i}+rand(0,1)\times (X-Z),i=1,2,\cdots ,n,\;X\in Z$$ (26)

Where *X*_*new*_ is the synthesized new sample, *Z*_*i*_ is the clustering center, *X* is the original sample with *Z*_*i*_ as the clustering center.

#### Experimental analysis

The data used in this paper comes from the written information statistics of various enterprises, and has been informed and agreed by the individual participants involved. All of them are adult employees, excluding minors. Meanwhile, the author was unable to identify the information of individual participants during or after all data collection periods. The employee datasets used are shown in Table 1. To verify the validity of the IFCM-SMOTE on the unbalanced datasets of resigned employees, the experiment divides the original samples into four types. The unbalance of the training samples is increasing in order, with a minimum of 3:1 and a maximum of 19:1.

**Table 1:** Sample information.

NO.	Sample size	Active employees	Resigned employees	Unbalance
Dataset-1	2000	1500	500	3:1
Dataset-2	2000	1600	400	4:1
Dataset-3	2000	1800	200	9:1
Dataset-4	2000	1900	100	19:1

The sample sets with four different unbalance were classified using SVM, SMOTE-SVM and IFCM-SMOTE-SVM, as shown in Fig 2. The comparison shows that the accuracy of the IFCM-SMOTE-SVM is better than that of the SMOTE-SVM and SVM on all four types of sample sets, and the accuracy gradually decreases as the unbalanced gets higher. From the above figure, we can also find that although the IFCM-SMOTE-SVM performs the best among the three algorithms, its accuracy only reaches about 80% when facing the employee datasets. The main reason for this is the influence of the SVM algorithm’s own characteristics, which leads to limited improvement of the final classification effect although the unbalanced datasets are first balanced by various methods artificially.

**Fig 2:** Comparison of accuracy of different methods.

### Prediction of employee turnover based on kernel space and IFCM-SMOTE-SVM

#### Modeling based on kernel space and SMOTE-SVM

*SMOTE-SVM with fusion kernel space*. Based on the above results, a kernel space-based SMOTE-SVM algorithm (KS-SMOTE-SVM) is proposed to optimize the accuracy of SVM for unbalanced data by directly oversampling minority instances in the feature space. Two instances *x*_*i*_ and *x*_*j*_ are redefined, and the distance *d*^*ϕ*^(*x*_*i*_,*x*_*j*_) between them after conversion to the high-dimensional feature space as:

$$d^{\phi }{\left(x_{i},x_{j}\right)}^{2}={\left\|\phi (x_{i})-\phi (x_{j})\right\|}^{2}=K(x_{i},x_{i})-2K(x_{i},x_{j})+K(x_{j},x_{j})$$ (27)

As with the SMOTE, a neighbor is randomly selected for each seed instance, which in turn generates a minority instance from both [40]. With the above, a set *S*^*syn*^ containing *P* data points is generated, where the *i*-th element $x_{i}^{pq}$ of *S*^*syn*^ is generated from the seed *x*^*p*^ and the neighbor *x*^*q*^, and all data points in *S*^*syn*^ are labeled with the minority class (+1). The kernel matrix *K* is decomposed as:

$$\begin{array}{c} K=\left[\begin{array}{cc} K^{1} & K^{2}\\ K^{2T} & K^{3} \end{array}\right]\\ K^{1}\in R^{N\times N}\;K_{ij}^{1}=K(x_{i},x_{j})\;x_{i},x_{j}\in S;\\ K^{2}\in R^{N\times P}\;K_{ij}^{2}=K(x_{i},x_{j}^{pq})\;x_{i}\in S,x_{j}^{pq}\in S^{syn};\\ K^{3}\in R^{P\times P}\;K_{ij}^{3}=K(x_{i}^{lm},x_{j}^{pq})\;x_{i}^{lm},x_{j}^{pq}\in S^{syn}. \end{array}$$ (28)

*K*^2^ is denoted as:

$$\begin{array}{l} K(x_{i},x_{j}^{pq})=\phi {\left(x_{i}\right)}^{T}\phi (x_{j}^{pq})\\ \;=\phi {\left(x_{i}\right)}^{T}[\phi (x_{p})+\delta^{pq}(\phi (x_{q})-\phi (x_{p}))]\\ \;=(1-\delta^{pq})K(x_{i},x_{p})+\delta^{pq}K(x_{i},x_{q}) \end{array}$$ (29)

The dot product *K*^3^ of $x_{i}^{lm}$ and $x_{j}^{pq}$ is given by the following equation:

$$\begin{array}{l} K(x_{i}^{lm},x_{j}^{pq})=\phi {\left(x_{i}^{lm}\right)}^{T}\phi (x_{j}^{pq})\\ \;=[\phi (x_{l})+\delta^{lm}{\left(\phi (x_{m})-\phi (x_{l})\right]}^{T}\times [\phi (x_{p})+\delta^{pq}(\phi (x_{q})-\phi (x_{p}))]\\ \;=(1-\delta^{pq})(1-\delta^{lm})K(x_{p},x_{l})+(1-\delta^{pq})(\delta^{lm})K(x_{p},x_{m})\\ \;+(\delta^{pq})(1-\delta^{lm})K(x_{q},x_{l})+(\delta^{pq})(\delta^{lm})K(x_{q},x_{m}) \end{array}$$ (30)

From Eqs (28), (29) and (30), it can be seen that the augmented kernel matrix *K* uses only the samples and kernel functions without an explicit mapping [41, 42]. Therefore, for SVM, any kernel function can be used, as long as it can eventually make the data set balanced. The KS-SMOTE-SVM proposed is well suited for use in the feature space of SVM classifiers. The Euclidean distance used in the algorithm is replaced by the feature space distance *D*(*x*_*i*_, *x*_*j*_) by Eq (27) and the kernel matrix is augmented using Eqs (28), (29) and (30) based on the selected seeds and neighbors.

RETRACTED

*Turnover prediction based on KS-SMOTE-SVM with fusion IFCM*. For an enterprise, the reasons why employee turnover often have commonality, which also makes the data of the employee turnover show the characteristics of clustering to certain key factors. Therefore, the IFCM-SMOTE-SVM of clustering and sampling is proposed in the previous paper, and the interpolation formula of the SMOTE is changed to:

$$X_{new}=Z_{i}+rand(0,1)\times (X-Z)$$ (26)

Where *Z*_*i*_ is the clustering center. Compared with the SMOTE, which randomly selects the center and generates new samples in the vicinity, the IFCM-SMOTE-SVM can generate more realistic and reliable samples. Therefore, the new kernel space-based SVM is proposed by combining the IFCM-SMOTE-SVM with the KS-SMOTE-SVM, named KS-IFCM-SMOTE-SVM, and bringing Eq (26) into Eq (29):

$$\begin{array}{l} K(x_{i},x_{j}^{pz})=\phi {\left(x_{i}\right)}^{T}\phi (x_{j}^{pz})\\ \;=\phi {\left(x_{i}\right)}^{T}[\phi (x_{z})+\delta^{pz}(\phi (x_{p})-\phi (x_{z}))]\\ \;=(1-\delta^{pz})K(x_{i},x_{p})+\delta^{pz}K(x_{i},x_{z}) \end{array}$$ (31)

Similarly, bringing Eq (26) into Eq (30) will result in a new kernel matrix *K*^3^. The above method can effectively solve the problem of synthesizing too much interference data by using the oversampling algorithm in the kernel space, which increases the reliability as well as the authenticity of the synthesized data.

### Experimental analysis

The datasets of employees of an enterprise within 2019 to 2022 are selected as the data. The datasets contain 2560 employees data, such as their age, gender, position, overtime, travel and other 35 columns of characteristic information. The ratio of the resigned employees to the active employees is 1:10, which satisfies the requirements of the unbalanced data. *TP* represents the samples in which active employees are correctly classified as active employees, *FN* represents the samples in which active employees are incorrectly classified as resigned employees, *FP* represents the samples in which resigned employees are incorrectly classified as active employees, and *TN* represents the samples in which resigned employees are correctly classified as resigned employees. Five evaluation criteria are calculated:

1. *Precision*, which indicates the proportion of- positive classes correctly predicted to the total samples:
$$Precision=\frac{TP}{TP+FP}$$ (32)
2. *Recall*, which indicating the proportion of positive classes correctly predicted to all positive classes:
$$Recall=\frac{TP}{TP+FN}$$ (33)
3. Overall Accuracy (*OA*), indicates the probability that the classification result of the sample is consistent with the data type:
$$OA=\frac{TP+TN}{TP+FP+FN+TN}$$ (34)
4. *F*-measure (*F*) is the summation of *Recall* and *Precision*:
$$F=\frac{(1+\beta^{2})\times recall\times precision}{\beta^{2}\times recall+precis}$$ (35)
5. G-mean (*G*) is the average performance in the correct positive and negative classes:
$$G_{mean}=\sqrt{\frac{TP}{TP+FP}\times \frac{TP}{TP+FN}}$$ (36)

In this paper, four models, SVM, SMOTE-SVM, KS-SMOTE-SVM and KS-IFCM-SMOTE-SVM, are compared to verify the effectiveness of the methods; 10 experiments were conducted on the employee datasets using each of the four models (Table 2). The traditional SVM performs the worst among the four, with the *Avg*. of *G* and *F* only 76.03% and 74.69%, respectively. SMOTE-SVM slightly improves the classification performance compared to the SVM, but it ends up being about 80%. After using the KS-SMOTE-SVM, the classification accuracy is significantly improved, with *G* and *F* reaching 91.50% and 90.71%, respectively. After combining with the IFCM clustering, the final improved algorithm (KS-IFCM-SMOTE-SVM) achieves the highest *Avg*. of *G* (95.93%) and *F* (95.33%). The experiments fully prove the effectiveness of this paper’s method for analyzing the turnover intention of enterprise employees.

RETRACTED

**Table 2:** Comparison of experimental results (%).

NO.	SVM		SMOTE-SVM		KS-SMOTE-SVM		KS-IFCM-SMOTE-SVM	
	*G*	*F*	*G*	*F*	*G*	*F*	*G*	*F*
1	76.03	74.69	81.15	80.78	91.04	90.49	96.07	95.61
2			80.40	79.04	90.43	90.33	95.23	94.10
3			82.07	81.65	93.49	91.98	95.30	94.56
4			82.26	81.10	92.21	91.49	96.51	95.91
5			79.01	78.94	90.91	90.04	96.14	95.24
6			77.21	76.24	90.23	89.71	95.21	94.92
7			79.48	79.05	90.56	89.67	95.00	94.51
8			76.97	76.26	91.88	91.02	96.56	95.99
9			81.15	80.91	92.86	91.81	96.98	96.69
10			80.92	80.63	91.36	90.52	96.33	95.80
*Avg*.	76.03	74.69	80.06	79.46	91.50	90.71	95.93	95.33

### Model optimization for employee turnover prediction

In the previous section, we found that the F-measure treats the loss of positive class misclassification and negative class misclassification cases equally. However, in the classification problem of unbalanced data, the importance of both is not the same, based on which the new evaluation index is proposed:

$$F_{t}=\frac{2TP_{t}}{2TP_{t}+(1+\beta )FN_{t}+(1-\beta )FP_{t}}\;,\beta \in [0,1)$$ (37)

In the above equation, *F*_*t*_ is the new evaluation index in round *t*, and *TP*_*t*_, *FN*_t_, *FP*_*t*_ are the classification corresponding to round *t*, respectively. To further verify the effectiveness of the algorithms on different types of datasets, we collected employee datasets from seven different types of enterprises, including different industries such as Internet, manufacturing, and e-commerce, as well as domestic and foreign enterprises. The performance of different models are compared, including KS-IFCM-SMOTE-SVM, KS-SMOTE-SVM, AdaBoost [43] and PIBoost [44] in integrated learning.

RETRACTED

From Fig 3, it can be found that the performance of KS-SMOTE-SVM on the datasets facing seven different types of enterprises have ups and downs, especially on the fifth dataset, the *Accuracy* is only 79%, which is obviously lower than expected. The *Accuracy* of AdaBoost and PIBoost algorithms are higher and lower than each other, where the *Accuracy* of AdaBoost on the third, fourth and seventh enterprise datasets are lower than those of KS-SMOTE-SVM, PIBoost is equal to KS-SMOTE-SVM on the second and sixth enterprise datasets, and the rest are slightly higher. The *Accuracy* of the KS-IFCM-SMOTE-SVM is better than the other three algorithms, which proves that the KS-IFCM-SMOTE-SVM obviously suppresses the overfitting problem of KS-SMOTE-SVM and integrated learning algorithms (AdaBoost and PIBoost), making it have good classification accuracy on different enterprise datasets.

**Fig 3:** Comparison of accuracy of different methods.

From Figs 4 and 5, it can be found that the results of using the KS-IFCM-SMOTE-SVM are better than the other three algorithms faced with employee datasets from different types of enterprises. From the *Accuracy* point of view, some employee datasets such as Dataset-B and Dataset-E obtained lower accuracy, but the *Accuracy* was substantially improved by the KS-IFCM-SMOTE-SVM. This is also due to the fact that the kernel space and FCM clustering focuses on the minority class of samples, i.e., resigned employees, which makes the KS-IFCM-SMOTE-SVM play a better classification effect when facing different types employee datasets. Looking at the *F* and *G*, we can see that the KS-IFCM-SMOTE-SVM performs the best on all datasets, with the *Avg*. of *F* reaching 89.62% and the *Avg*. of *G* reaching 89.05%. The algorithm can guarantee the classification effectiveness when facing different types employee datasets, which greatly improves the classification effect of SVM on unbalanced data and optimizes the prediction model for employee turnover in different industries.

**Fig 4:** Comparison of F-measure of different methods.

**Fig 5:** Comparison of G-mean of different methods.

## Conclusion

The SMOTE oversampling method is introduced to improve the deficiency of SVM for generated samples without misclassification cost in the classification process. The improved FCM clustering algorithm is proposed to generate new samples in combination with the SMOTE, which greatly reduces the chances of noisy data generation. The KS-IFCM-SMOTE-SVM based on the kernel space is obtained by using the kernel function of SVM to transform the data into the high-dimensional feature space before clustering and sampling, and the method is experimentally demonstrated to have a great improvement on the classification accuracy of SVM.

1. For the characteristics of the unbalanced data in the employee datasets of enterprises, the oversampling-based SMOTE is introduced in SVM to improve the unbalanced nature of the datasets. Weighting of the synthetic samples to address the drawback that the SVM does not distinguish the cost of misclassification further improves the accuracy of the SMOTE-SVM.
2. The improved FCM clustering algorithm based on SMOTE (IFCM-SMOTE-SVM) is proposed. Combined with the SMOTE oversampling algorithm, the datasets of resigned employees are clustered first and then sampled, thus making the synthetic data have higher accuracy and realism. The experimental comparison of the unbalanced data proves that the algorithm has a better improvement on the classification accuracy of SVM.
3. The kernel space-based SMOTE-SVM (KS-SMOTE-SVM) is proposed after finding that SMOTE is overly dependent on specific data distribution features. Combined with the IFCM-SMOTE-SVM, the original dataset is converted to the high-dimensional kernel space before clustering and oversampling, and then finally classified by SVM, named KS-IFCM-SMOTE-SVM. The experimental comparison shows that the algorithm has a significant improvement in the classification accuracy.
4. The new evaluation metric is constructed to verify the performance of the KS-IFCM-SMOTE-SVM in the face of different datasets. Comparative experiments are conducted on the employee datasets from different types of enterprises, and it is demonstrated that KS-IFCM-SMOTE-SVM has a significant improvement in Accuracy, F-measure and G-mean on different datasets, which can optimize the prediction model for employee turnover in different industries.
